# Insights on the epigenetic mechanisms underlying pulmonary arterial hypertension

**DOI:** 10.1590/1414-431X20187437

**Published:** 2018-10-18

**Authors:** R.C.P. Luna, Y. de Oliveira, J.V.C. Lisboa, T.R. Chaves, T.A.M. de Araújo, E.E. de Sousa, M. Miranda, L. Pirola, V.A. Braga, J.L. de Brito Alves

**Affiliations:** 1 Departamento de Nutrição, Centro de Ciências da Saúde, Universidade Federal da Paraíba, João Pessoa, PB, Brasil; 2 INSERM U1060, Lyon 1 University, Oullins, France; 3 Departamento de Biotecnologia, Centro de Biotecnologia, Universidade Federal da Paraíba, João Pessoa, PB, Brasil

**Keywords:** Epigenetic, Pulmonary arterial hypertension, DNA Methylation, Histone acetylation, miRNAs

## Abstract

Pulmonary arterial hypertension (PAH), characterized by localized increased arterial blood pressure in the lungs, is a slow developing long-term disease that can be fatal. PAH is characterized by inflammation, vascular tone imbalance, pathological pulmonary vascular remodeling, and right-sided heart failure. Current treatments for PAH are palliative and development of new therapies is necessary. Recent and relevant studies have demonstrated that epigenetic processes may exert key influences on the pathogenesis of PAH and may be promising therapeutic targets in the prevention and/or cure of this condition. The aim of the present mini-review is to summarize the occurrence of epigenetic-based mechanisms in the context of PAH physiopathology, focusing on the roles of DNA methylation, histone post-translational modifications and non-coding RNAs. We also discuss the potential of epigenetic-based therapies for PAH.

## Introduction

Pulmonary arterial hypertension (PAH) is a severe and multifactorial disease with a high incidence worldwide (1). The incidence of PAH ranges from 2 to 7.6 cases per million adults per year, while its prevalence varies from 11 to 26 cases per million adults (2 [Bibr B03]–4). PAH is defined as mean pulmonary artery pressure above 25 mmHg and pulmonary artery occlusion pressure lower than 15 mmHg. PAH is categorized as idiopathic (iPAH), inheritable, toxin- or drug-induced, or linked to other pathological conditions, such as human immunodeficiency virus (HIV) infection, portal hypertension, congenital heart disease, or schistosomiasis.

Despite considerable advances in the understanding of the pathophysiology, diagnosis, and treatment of PAH, the molecular mechanisms underlying the PAH remain unclear. Physiopathological alterations in patients with PAH have been related to age, sex, and the presence of co-morbidities, and they collectively contribute to the patient’s survival (5).

Recent findings have indicated that epigenetic modifications may be associated to the pathogenesis of PAH (6,7). Evidence shows that DNA methylation, histone post-translational modifications, and micro-RNA (miRNA)-associated gene silencing are found in both human and animal models of PAH (8). For example, histone deacetylation and miRNAs dysregulation are observed in the hyper-proliferation of pulmonary artery smooth muscle cells (PASMCs) (7). Additionally, DNA cytosine methylation can silence genes through a process that leads to the compaction of the chromatin structure or by acting directly on the DNA promoter region (9). Accordingly, previous studies have shown that DNA hypermethylation in the superoxide dismutase 2 (SOD2) genomic region can lead to reduced SOD2 expression in PASMCs and contribute to hyper-proliferation of these cells in PAH patients (10,11).

To highlight these new insights, we discuss here the current advances in our understanding of how epigenetic dysregulations are associated with PAH, and how targeting such defects may open the way to innovative therapies.

## Physiopathology of PAH

The pathogenesis of PAH is complex and still has not been completely elucidated. Thus, a better understanding of disease pathogenesis is essential to identify new targets for therapy. PAH is characterized by augmented vasoconstriction, vascular obstruction, inflammation, fibrosis, vascular stiffening, endothelial dysfunction, and right ventricular failure (12).

Abnormal pulmonary vascular reorganization, including excessive vascular proliferation and resistance to apoptosis of pulmonary artery smooth muscle cells (PASMCs) within the vascular wall, contributes to reduction of arterial compliance and increased vascular resistance and blood pressure, resulting in right-side heart failure and premature death. Patients with PAH exhibit multiple nonspecific symptoms, with fatigue, weakness, dizziness, and progressive shortness of breath on exertion being often reported by patients (12).

Several underlying mechanisms leading to excessive proliferative and reduced apoptosis in PASMCs have been previously elucidated. For example, increased cytosolic calcium via activation of store-operated Ca^+2^ channels or down-regulation of voltage-gated potassium channels, such as Kv1.5, facilitate the contractile, hyperproliferative, and anti-apoptotic phenotype of PASMCs in PAH (13). In addition, mitochondrial dysfunction, including a metabolic shift from glucose oxidation toward uncoupled aerobic glycolysis, unregulated glycolysis and mitochondrial fragmentation, and membrane hyperpolarization support rapid proliferation and resistance to apoptosis in PASMCs (14).

The importance of cardiac dysfunction in the right ventricle (RV) in PAH is attracting increasing interest due to its critical association with the morbidity and mortality of the disease. An alteration of the autonomic balance, characterized in particular by a dysfunction of cardiac variability and a reduced parasympathetic sensitivity (15), is associated with a poor prognosis in PAH patients (16). In addition, hyperactivation of the sympathetic nervous system has been demonstrated in clinical and experimental studies as one of the main factors associated with autonomic dysfunction in PAH (17). Sympathetic hyperactivation is characterized by an increase in the intensity and frequency of electrical depolarizations of the sympathetic nerve and by an increase in the plasmatic levels of catecholamines, promoting constriction of peripheral blood vessels, increased vascular resistance, and consequent increase in baseline blood pressure levels. Because of this, circulating catecholamines are augmented in PAH patients with RV failure (18). In addition, endothelial dysfunction has been observed in the development and progression of vascular pathology in PAH. Patients with PAH exhibit pulmonary endothelial dysfunction and decreased nitric oxide (NO) bioavailability, characterized by a reduced endothelial NO synthase (eNOS) expression, and low synthesis and release of NO, the main vasodilator substance produced by the endothelium of the pulmonary vessels (19).

## Epigenetic mechanisms

The term epigenetics was originally proposed by Conrad Waddington (1942), to describe of the occurrence of biologically relevant processes resulting from the interplay between the genome (and its functional units: the genes) and the environment, which lead to different phenotypic manifestations (20). In other words, epigenetics refers to the manifestation or transmission of specific characters whose information is not contained within the DNA 4 base code. The main epigenetic mechanisms that in mammalian cells contribute to the regulation of gene expression include DNA methylation, histone post-translational modifications (such as methylation, acetylation, phosphorylation), and ubiquitination (21). More recently, non-coding RNAs have been also demonstrated to be involved in the post-transcriptional regulation of gene expression in multicellular organisms (22).

Cytosine DNA methylation, taking place on cytosines within the CpG dinucleotide sequence, is a process catalyzed by DNA methyltransferases (DNMTs) enzymes, and is a key epigenetic mechanism associated to gene expression modulation. It has been proposed that CpG islands, found in gene promoter and other genomic regulatory relevant regions, when hyper-methylated, lead to gene silencing (23).

In addition to cytosine methylation, post-translational modifications taking place in the histone subunits composing the histone octamer also contribute to the definition of gene expression patterns. Histones are highly evolutionarily conserved proteins, which are essential in the composition of the nucleosome of eukaryotic chromatin. The histone octamer is composed of dimers of each of four central core histones (H2A, H2B, H3, and H4) (24). DNA is wrapped around the histone octamer, and collectively, the histone octamer and the associated DNA form the nucleosome: the basic repeating unit of chromatin. Nucleosomes are “sealed” externally by histone H1. Histone acetylation is a reversible and dynamic epigenetic mechanism determined by the balance between histone acetyltransferases (HATs) and histone deacetylases (HDACs). In general, the deacetylation process is associated with condensed chromatin (heterochromatin) and transcriptional repression.

miRNAs act as important regulators of gene expression as part of the epigenetic machinery. Distinct biotypes of extracellular RNA have been detected in human circulation in the form of small regulatory non-coding RNAs (sRNAs). Typically, sRNAs range from 15 to 200 nucleotides, with miRNAs being the most widely studied in mammals (25).

### DNA methylation

DNA methylation, one of the most widely studied epigenetic mechanisms, is a biochemical reaction of covalent addition of a methyl (CH_3_) group to cytosine residues, usually within CG dinucleotides enriched in genomic regions named CpG islands. DNA methylation is accomplished by DNMTs (26). DNMTs are thus involved in *de novo* DNA methylation and maintenance of genome methylation (27). Four main variants of DNMTs are found in humans, namely DNMT1, DNMT3A, DNMT3B, and DNMT3L, to mediate the methylation process. DNMT1 serves to maintain the existing methylation patterns. DNMT3A and DNMT3B, on the other hand, regulate the *de novo* methylation, while DNMT3L functions as a unique co-factor in the methylation of imprinted genes in gametic cells (28). In general, DNA methylation promotes condensation of chromatin structure, leading to the silencing or suppression of gene expression.

### Histone post-translational modifications (PTMs)

Enzyme-mediated acetylations and methylations occurring on histones do not constitute the only possible PTMs taking place on histones. Indeed, while acetylation and methylation are the most studied phenomena, histones are also submitted to phosphorylation, sumoylation, ubiquitination, and ribosylation. These modifications appear in specific amino acids: acetylation on lysines (K), methylation on lysines and arginines (R), phosphorylation on serines (S) and threonines (T), ubiquitylation, and sumoylation and ribosylation on lysines (29).

Collectively, these PTMs have an influence on the structure and the level of condensation of the chromatin and are part of a “histone code” at the basis of gene regulation (30). Histone acetylation and deacetylation play an important part in the nucleosome modifications process. They are caused by acetylation and deacetylation complexes and yield a covalent modification of the nucleosome by changing the histones tail conformation by adding and removing acetyl groups from the amino termini of the four core histones. Acetylation and deacetylation are mediated by HATs and HDACs, respectively. Acetylation, mediated by HATs, is the reversible reaction where one acetyl group is transferred from an AcetylCoA to the lysine e-amino group. The removal of the acetyl moiety is made by HDACs, with the production of H_2_O. Acetylation is mostly linked to transcriptional activation.

#### Histone acetyltransferases (HATs)

HATs can be separated into two groups: Type A located in the nucleus and acetylating histones, in the timing needed for transcriptional activation, and Type B located in the cytoplasm, responsible for histone acetylation during replication and before the chromatin’s assemblage. HATs are responsible for histone acetylation, but can also acetylate other non-histones proteins in various nuclear and cytoplasmic pathways (31). Among the most active HATs in mammals are found cAMP response-element binding protein (CREB) binding protein (CBP), p300, p300/CREB binding protein-associated factor (PCAF), and HIV Tat interactive 60-kDa protein (Tip60). Specific HATs recruited by steroid receptors exist also, such as steroid receptor coactivators 1 and 3 (SRC-1 and -3) (31).

#### Histone deacetylases (HDACs)

HDAC activity was first discovered in yeast. The use of trapoxin, an antitumor cyclic tetrapeptide, showed increased histone acetylation, and led to the identification of the protein responsible: the first histone deacetylase. HDACs can be separated into 3 different groups based on their similarities with the yeast histone deacetylase: *i*) class I HDACs (HDAC 1, 2, 3, and 8) located in the nucleus and similar to the yeast RPD3 protein, *ii*) class II HDACs (HDACs 4, 5, 6, 7, 9, and 10) present in both nucleus and cytoplasm and similar to the yeast HDA1 protein, and *iii*) class III HDACs (Sirtuins 1-7) analogous to the yeast Sir2 proteins. HDACs play a major role adjusting acetylation and deacetylation levels of chromatin (32).

#### Sirtuins

A particular HDAC class, sirtuins are a specific class of HDACs that are dependent on nicotine adenine dinucleotide (NAD^+^) for their activity. They regulate numerous activities like cell division, transcription, metabolism, stress damage, and aging. Seven sirtuins exist with specific locations in the cell: Sirt1, 6 and 7 are in the nucleus, Sirt2 in the cytosol, and Sirts3, 4, and 5 in the mitochondria (33).

#### Histone methylation

Histone methylation is a transcriptionally promoting, or repressing PTM. Methylation concerns lysine and arginine residues. Contrary to acetylation, methylation marks can be multiple. Arginines can be unmethylated, monomethylated, or dimethylated. Furthermore, arginine dimethylation can generate asymmetric dimethylarginines and symmetric dimethylarginines (34). Each lysine residue can be mono-, di- or trimethylated. Histone lysine methylation appears to occur preferentially on H3 and H4. Methylation is catalyzed by histone methyltransferases (HMTs). The methyl-transfer reaction uses s-adenosylmethionine (SAM) as a methyl donor; in the same way, HATs use acetyl groups derived from acetylCoA (35). Histone methylation is a more permanent mark than acetylation. Indeed, histone acetylation can occur all along the cell cycle whereas histone methylation is associated to heterochromatin formation with methylation levels peaking in the G2 phase following DNA replication and histone re-deposition.

### Histone methyltransferases

Methylation is orchestrated by HMTs. HMTs responsible for the arginine methylation are called protein arginine methyltransferases (PRMTs), and 11 isoforms, divided into 3 groups, type I, II, and III, exist in mammals (36). In the same way, methyltransferases responsible for the specific methylation of lysines are called lysine methyltransferases (KMTs) and are divided into six families based on the structural particularity of their catalytic SET domain (37).

#### Histone demethylases (HDMs)

As mentioned above, methylation was thought to be an irreversible/permanent epigenetic mark, a belief derived from the high thermodynamic stability of the N–CH3 bond. The understanding of the methylation regulation changed with the discovery of one histone demethylase, LSD1. Later, many enzymes regulating histone demethylation were discovered. Demethylation mechanisms differ depending on the amino acid carrying the methylation, lysine or arginine, and the methylation profile, one to three methyl groups. Two types of histone demethylases exist: a flavin adenine dinucleotide (FAD)-dependent amine oxidase and Fe (II) and α-ketoglutarate-dependent dioxygenase. For the first type, which includes the amine oxidase LSD1, demethylation requires FAD as a cofactor during the removal of a methyl group and produces hydrogen peroxide and formaldehyde (38). In the second type, demethylation by an iron-dependent and alpha-ketoglutarate-dependent oxidation reaction mechanism as found in yeast is conserved in eukaryotes. The enzyme, containing a JmjC domain, is capable of demethylating DNA, producing formaldehyde and succinate as reaction products.

### Ubiquitination

The ubiquitin-proteasome system (UPS), a major protein quality and quantity control system, is a post-translational mechanism particularly interesting from both structural and functional viewpoints, involved in the regulation of many cellular processes including protein degradation, gene expression, signaling transduction, and apoptosis (39). Ubiquitin is a 76-amino acid protein ubiquitously distributed in all tissues of eukaryotic organisms. In this process, the C-terminal carboxyl group of ubiquitin becomes attached to the ε-amine of a lysine residue of the substrate protein through an isopeptide bond. Ubiquitination is a multi-step and reversible process that involves a cascade of three essential enzymes: ubiquitin-activating enzymes (E1), ubiquitin-conjugating enzymes (E2), and ubiquitin ligases (E3). E1 and E2 enzymes prepare ubiquitin for conjugation. E3 enzymes recognize the specific substrate and catalyze the transfer of activated ubiquitin to the substrate. Recently, the activity of an E4 enzyme has been described as catalyst for the conjugation of additional ubiquitin monomers to form polyubiquitin chains, usually through lysine 48 (K48) linkages (40). The processes of ubiquitination and de-ubiquitination are controlled with high specificity; however, dysfunctions in this complex are implicated in many human diseases (40).

### Non-coding RNAs

Non-coding RNAs (ncRNAs) are the transcription products of non-coding genes (i.e., lacking the ability to be translated into proteins). Non-coding RNAs include tRNAs, rRNAs, snoRNAs, microRNAs, siRNAs, snRNAs, exRNAs, piRNAs, and scaRNAs and the long ncRNAs (41). The development of next-generation sequencing technologies identified thousands of ncRNAs. These ncRNAs can be divided into two main classes: small ncRNAs (<200 nucleotides long), which include microRNAs (miRNAs), piwi-interacting RNAs (piRNAs), and small-interfering RNAs (siRNA), their main function is to modulate gene expression through direct binding to coding or non-coding sequences of mRNAs; and long-non-coding RNAs (lncRNAs) (>200 nucleotides long), which include natural antisense transcripts, small nucleolar RNAs (snRNA), and other types of lncRNAs. Specifically, miRNAs are post-transcriptional regulators, piRNAs can modulate DNA methylation and transposon repression, and siRNAs are known as short interfering RNA or silencing RNA, similar to miRNA, and operating through the RNA interference (RNAi) pathway. In addition, lncRNAs are epigenetic regulators of transcription, the snRNAs are mainly involved in nucleotide modification of ribosomal RNA, and circular RNAs (circRNAs) are miRNA sponging and RNA polymerase II regulators (41).

## DNA methylation and PAH

It has been suggested that down-regulation of SOD2 can activate the hypoxia-inducible factor 1 alpha (HIF-1α) and create a pseudo-hypoxic environment favorable to a glycolytic metabolic state and harmful to oxidative metabolism in PASMCs of fawn-hooded rats. Studies have shown that the hypermethylation mechanisms in CpG islands mediated by DNMT1 and DNMT3B contribute to the down-regulation of SOD2 mRNA in PAH (10,11). These alterations may be able to enhance the proliferation of the PASMCs in PAH.

It is reasonable to suggest that DNA methyltransferase inhibitors, by decreasing DNA methylation on the SOD2 gene locus and consequently favoring the SOD2 gene and protein expression, may be able to alleviate PASMCs proliferation and consequently SOD2 down-regulation in PAH. Studies conducted on the fawn-hooded rat, which develops PAH spontaneously, have demonstrated that treatment with 5-aza-2′-deoxycytidine (a DNMT inhibitor) or with MnTBAP (a mimetic of SOD2), at a dose of 10 mg/kg for 2 weeks, was capable of increasing SOD2 expression while reducing the proliferative state of PASMCs, resulting in alleviated pulmonary arterial hypertension (10,42). Therefore, the understanding of the relationship between DNA methylation and SOD2 expression might be an important step towards better elucidation of the pathophysiologic alterations in PAH and possibly the development of a new therapeutic target for this disease. In addition, future studies will need to examine whether HIF-1α inhibitors are able to exhibit beneficial results under the PAH condition.

Heritable forms of PAH represent approximately 6–10% of all PAH. From a genetic basis, the most recognized genetic variants linked with PAH occur in type 2 bone morphogenetic protein receptor 2 (BMPR2). BMPR2 mutations are responsible for the etiology of approximately 80% of patients with familial PAH and 30% idiopathic PAH (43,44). Thus, a BMPR2 gene mutation increases the chance of developing PAH. Another important point is that BMPR2 mutations are considered to be permissive of disease and require additional genetic, epigenetic, or environmental influences for the development of PAH in individuals with mutations (2). Low BMPR2 protein expression or impaired BMPR2 signaling in lung tissue and endothelial cells have been shown to promote accelerated cell proliferation and facilitate the development of PAH (45). A study analyzing whether alterations in DNA methylation pattern could be associated to BMPR2 mutations in 28 patients with iPAH and 27 patients diagnosed with PAH associated with other diseases found no difference in the methylation CpG islands of BMPR2 promoter region between the PAH patients and healthy control subjects (46). On the contrary, a recent study demonstrated that hypermethylation in the BMPR2 promoter does occur in patients with heritable pulmonary arterial hypertension, resulting in down-regulation of BMPR2 expression (47). Together, these findings show that DNA methylation mechanisms involved in PAH are complex and unmistakable, take place on multiple genes, and are not the only mechanisms associated with all forms of PAH. Therefore, there is a need to further explore cytosine methylation mechanisms in PAH as potential targets for future new therapies.

## Histone acetylation and PAH

Recent findings have shown that histone acetylation is likewise important in cardiopulmonary remodeling. However, a satisfactory understanding of the mechanism(s) by which histone acetylation dysregulation impacts pulmonary remodeling in PAH will require more research (48).

Talati and colleagues observed that histone H1 expression was reduced in the pulmonary artery and PASMCs of patients with iPAH. The authors suggested that the reduced H1 expression could contribute to a less condensed chromatin pattern and consequently facilitate the activation of transcriptional pathways contributing to PAH (49).

Histone acetylated lysines, under the control of the opposite action of HATs and HDACs, are recognized by bromodomain and extra-terminal (BET) proteins. BET proteins binding to acetylated histones promote transcriptional elongation and upregulation of genes involved in cell proliferation, apoptosis, and inflammation (50).

HAT activity and the HAT:HDAC ratio have been reported to significantly increase in the lungs of patients with iHAP. High HAT activity has also been linked to elevated expression levels of BET proteins under the PAH condition (50). BET proteins are essential for the activation of inflammatory transcription nuclear factor kappa-light-chain-enhancer of activated B cells (NF-κB), up-regulation of pro-inflammatory genes, alteration in the proliferation/remodeling of vascular endothelial cells, and appear to play a direct role in the PAH pathogenesis (51).

Interestingly, the inhibition of BETs in primary human pulmonary microvascular endothelial cells (HPMECs) induced a significant reduction in inflammation and pulmonary remodeling (50). Thus, BET inhibition is another promising target for future therapies against PAH.

An excessive accumulation of reactive oxygen species (ROS), increased expression of NADPH oxidase and down-regulation of antioxidant enzymes also has been reported in PAH. In addition, a defect of the histone acetylation process has been observed in oxidative stress pathways (52). Of note, Chen and colleagues found that HDAC inhibitors potently reduce transcription of NADPH oxidases and ROS production and ameliorate PAH in monocrotaline (MCT) rat model (53).

SOD3, an extracellular isoform of the superoxide dismutase, is an important antioxidant enzyme in the vasculature system. Experimental and clinical studies have reported that SOD3 expression is reduced in PAH (54,55). Nozik-Grayck and colleagues investigated whether aberrant DNA methylation and/or histone deacetylation could be the reason for reduced SOD3 expression in iPAH. The authors demonstrated that DNA methylation was not responsible for SOD3 down-regulation in PASMC of iPAH patients (56). Additionally, HDAC and HAT activities were similar in the PASMC of healthy subjects and iPAH patients. However, it was observed that treatment with selective class I HDAC inhibitors increased SOD3 expression in PASMC of iPAH patients. Thus, targeting of HDACs with HDAC inhibitors (HDACi) could represent a potential therapeutic approach for iPAH, at least in part, because of the HDACi-induced SOD3 expression in PASMC (56).

Similarly, treatment with valproic acid, a class I HDAC inhibitor, at 300 mg/kg during 5 weeks, has also been shown to reverse the development of severe pulmonary arterial hypertension in MCT and chronic hypoxia rat models (57). Based on those findings, it is reasonable to propose that HDACi may be useful in the treatment of PAH.

## Ubiquitination and proteasome activity in PAH

Although the precise mechanism(s) still need to be fully elucidated, recent studies have demonstrated that the ubiquitin-proteasome complex might be involved in PASMCs proliferation in PAH, and consequently might represent a new target for treatment of PAH (58,59). It has been demonstrated that intersectin-1s (ITSN-1s), a multidomain adaptor protein regulating endocytosis, cytoskeletal rearrangements, cell signaling, and the ubiquitination process is reduced in PAH (60).

In addition, it has been shown that proteasome inhibitors can suppress the growth of pulmonary PASMCs and consequently might be useful for treating PAH (59). Using bortezomib (BTZ), the first proteasome inhibitor to be approved by the FDA, pulmonary vascular remodeling was successfully reversed in PAH rats (61). However, BTZ caused cardiac apoptosis in both the RV and the left ventricle (LV) in PAH rats, limiting their clinical applicability. Carfilzomib (CFZ), another proteasome inhibitor, administration in combination with vasodilators and cardioprotectants has been demonstrated as an effective therapy for the treatment of PAH. CFZ was more effective in killing human pulmonary vascular cells than BTZ (62). The mechanism of proteasome inhibition involves the active role of ubiquitin in promoting apoptosis as well as autophagy in PASMCs in PAH (62).

## Role of non-coding RNAs in PAH

Traditionally, studies of gene expression and epigenetics have been focused on proteins that act as transcription factors and enzymes modulating histones post-translational modifications and DNA methylation. More recently, cumulative evidence suggested the involvement of RNA molecules as an additional regulatory player contributing to the determination of chromatin structure.

It is well known that the primary cellular mechanism underlying vascular remodeling under the PAH condition is the excessive proliferation of PASMCs (63). It has also been suggested that PASMC proliferation may be associated with aberrant microRNA signatures, which might provide some insights into the pathogenesis of PAH (64,65).

miRNAs have been described as playing essential roles in genic modulation and various cellular process, such as proliferation, differentiation, and apoptosis (66). There is growing evidence that a set of miRNAs is involved in the process of angiogenesis and vascular remodeling, which are prognostic events in the pathogenesis of PAH (66–68). Thus, investigation and understanding of the miRNA dysregulation events taking place in PAH may lead to the uncovering of useful biomarkers and/or new therapeutic targets for the treatment of PAH (69).

Previous reports have shown that a number of miRNAs, such as miR21, miR-103/107, miR-140-5p, miR-199a-5p, miR-223, let-7a-5p, miR-26b-5p, miR-27b-3p, miR-199a-3p, and miR-656, act together to control PASMCs proliferation in PAH both in cell culture and rat models (Table 1).

**Table 1.** Non-coding RNAs involved in pulmonary arterial hypertension (PAH) development.

miRNAs	Expression in PAH	Primary endpoint observed	Models	Reference
miR-21	up-regulated	Increased PASMCs proliferation.	PASMCs culture from PAH patients.	Sarkar et al., 2010 70
miR-98	down-regulated	Linked with augmented ET-1.	Pulmonary artery endothelial cell culture of PAH patients and hypoxia-induced PAH in rat.	Kang et al., 2016 71
miR-103/107	down-regulated	Related to activation of HIF-1β signaling pathways, enhanced proliferation of PASMCs and vascular remodeling in PAH.	Hypoxia-induced PAH in rat.	Deng et al., 2016 72
miR-135a	up-regulated	High right ventricular systolic pressure linked to BMPR2 down-expression in lung.	Experimental mouse model.	Lee and Park, 2017 75
miR-140	up-regulated	Linked to reduced MFN1 expression in hypertrophic right ventricles from PAH rats.	Sugen-5416 injection plus hypoxia exposure-induced PAH rats.	Joshi et al., 2016 76
miR-140-5p	down-regulated	High PASMC proliferation dependent of SMURF1 pathways.	PASMCs culture from PAH patients.Monocrotaline-induced PAH in rat.	Rothman et al., 2016 77; Zhang and Xu, 2016 78
miR-204	down-regulated	RUNX2 overexpression and HIF-1α activation linked to PASMC proliferation in PAH.	PASMCs culture from PAH patients, human PAH lung and Sugen/hypoxia-induced PAH in rats.	Ruffenach et al., 2016 79
miR-223	down-regulated	miR-223 overexpression in hypoxia-induced PAH model, it is associated with attenuation in pulmonary arterial pressure.	Human PAH lung, distal pulmonary arterioles and PASMCs culture.	Meloche et al., 2015 82; Smith et al., 2015 81
miR-210	up-regulated	Induce PASMC proliferation HIF-1α dependent.	PASMCs culture and hypoxia-induced PAH in rat.	Gou et al., 2012 87
miR-199a-5p	up-regulated	Associated with lower level of oxide nitric in PAH.	PAH in rat models and PASMCs culture from PAH patients.	Liu et al., 2016 86
let-7a-5p,miR-26b-5p, miR-27b-3p, miR-199a-3p, and miR-656	up-regulated	Activated a wide-ranging of Wnt/β-catenin pathway, leading to vascular remodeling and complications in PAH.	Lung tissues from IPAH patients.	Wu et al., 2016 88

miRNA, miR-: micro-RNAs; PASMC: pulmonary artery smooth muscle cells.

MiR-21 expression has been shown to be augmented in hypoxia-induced PASMCs proliferation. Interestingly, when miR-21 is inhibited (anti-miR-21), cell proliferation is reduced in primary PASMCs cell cultures derived from patients with PAH, demonstrating that miR-21 plays an important function in PASMCs proliferation (70).

Hypoxia, a common stimulus for PAH, decreased miR-98 expression and augmented endothelin-1 (ET-1) levels in the lungs of mice. Pharmacological activation of peroxisome proliferator-activated gamma receptor (PPARγ) with rosiglitazone restored miR-98 levels, reducing ET-1 and the proliferation of pulmonary artery endothelial cells (71).

Recently, Deng and colleagues demonstrated that miR-103/107 also regulates the proliferation of PASMCs under PAH conditions in a rat model. Down-regulation of miR-103/107 was linked to activation of HIF-1β-dependent signaling pathways, which resulted in enhanced proliferation of PASMCs and vascular remodeling in PAH (72).

Regarding the role of miR-127a, it has been demonstrated that miR-127a is up-regulated in the lungs of a hypoxia-induced PAH experimental model. This up-regulation was linked to reduced PPAR gamma levels and pulmonary artery endothelial cell hyper-proliferation (73). Recently, the mechanism by which miR-127a/b is linked to PPARγ down-regulation and PASMCs hyper-proliferation has been better elucidated. It was found that ET-1 causes NF-κB pathway activation and subsequent miR-127a/b up-regulation, which leads to post-transcriptional suppression of PPARγ expression and controls the proliferation of PASMCs (74).

MicroRNA-135a has also been associated with PAH. miR-135a levels were found to be up-regulated in the lung of an experimental mouse model displaying PAH (75). A recent study investigated whether miR-135a could influence BMPR2 expression in an experimental mouse model of PAH. Lee and colleagues demonstrated that miR-135a was significantly increased and BMPR2 significantly decreased, suggesting that BMPR2 may be an important target of miR135a in PAH. Additionally, the study demonstrated that treatment with antagomiR-135a for three weeks, improved right ventricular systolic pressure and right ventricular hypertrophy and augmented both mRNA and protein expression of BMPR2 (75).

Hypoxia leads to upregulation of mitofusin 1 (MFN1), a mitochondrial fusion protein, both *in vivo* and *in vitro*. MFN1 is involved in hypoxia-induced PASMCs proliferation in PAH (76). Regarding the role of miR-140 on MFN1 expression in PAH, up-regulation of miR-140 has been shown to be linked to reduced MFN1 expression in the hypertrophic right ventricles of PAH rats (76).

Previous reports have demonstrated that the expression of miR-140-5p was reduced in experimental models and in patients with PAH (77,78). Some authors have proposed that SMAD-specific E3 ubiquitin protein ligase 1 (SMURF1) could be a key regulator for miR-140-5p targets and bone morphogenetic protein (BMP) signaling. This indicates that reduced miR-140-5p expression is associated to increased pulmonary vascular SMURF1 protein expression and reduced BMP signaling in patients with PAH and that inhibition of SMURF1 provides a potential mechanism by which BMP signaling may be augmented for therapeutic benefit (77).

Interestingly, Dnmt1 is also a potential target of miR-140-5p. Reduced miR-140-5p contributes, at least in part, to Dnmt1 overexpression and consequently to down-regulation of SOD2 expression and hyper-proliferation of PASMCs in PAH. Furthermore, increased miR-140-5p inhibits proliferation and promotes apoptosis and differentiation of PASMCs under hypoxic conditions (78).

MiR-204 attenuation has been shown to promote up-regulation and sustained expression of the Runt-related transcription factor 2 (RUNX2) and HIF1α in PAH. These alterations are associated with aberrant proliferation and resistance to apoptosis in PASMCs in a subset of patients with PAH (79).

MiR-223 has been primarily described in hematopoietic cells and some tumoral processes (80). Recent studies, however, have also investigated its function in PAH (81). Expression of miR-223 is down-regulated in the human PAH lung, distal pulmonary arterioles, and PASMCs (82). Similarly, in the hypoxia-induced PAH model, miR-223 is down-regulated in PASMCs. When miR-223 was over-expressed in hypoxia-induced PAH model, there was attenuation in pulmonary arterial pressure (81,82).

Mechanistically, it has been proposed that miR-223 overexpression could inhibit key regulators of actin dynamics and cell proliferation, such as myosin phosphatase (MYPT1) and RhoB, attenuating vascular remodeling and PAH (67). In agreement with this, recent studies have demonstrated that inhibition of the Rho family protein with the selective Rho inhibitors tipifarnib or fasudil is capable of attenuating ventricular remodeling (83) and preventing development of hypoxia-induced PAH (84).

Shi and colleagues demonstrated that the miR-223 down-regulation observed in PAH is linked to increased expression of the insulin-like growth factor-I receptor (IGF-IR) in human pulmonary hypertension. On the other hand, when miR-223 is overexpressed, or upon pharmacological inhibition of IGF-IR, right-ventricular hypertrophy is attenuated and right heart function is improved under hypoxia (85). Together, these findings show that miR-223 can act in modulating different signaling pathways in PAH.

miRNA-199a-5p is another non-coding RNA that plays important roles in PAH (86). While multiple studies have shown that non-coding RNAs are mostly down-regulated in PAH, a recent study has demonstrated that the expression of miR-199a-5p and miR-210 are significantly increased under PAH (86,87). miR-199a-5p is associated with lower levels of NO in PAH and administration of anti-miR-199a-5p restored increased levels of NO and improved pulmonary artery pressure and right ventricular hypertrophy (86).

In a study on microRNA abundance in end-stage iPAH, five miRNAs (let-7a-5p, miR-26b-5p, miR-27b-3p, miR-199a-3p, and miR-656) were found to be significantly up-regulated in lung tissues (88). In this study, the authors showed that the upregulation of these miRNAs activated the Wnt / β-catenin pathway, leading to vascular remodeling and complications of iPAH.

Taken together, these findings have demonstrated that miRNAs could become important biomarkers for the diagnosis of severity and prognosis of PAH. miRNAs also represent a promising target in clinical strategies aiming at improving the prevention and therapeutic treatment of PAH. However, it should be noted that the significance of miRNA expression must be interpreted cautiously depending on the expression site or cells.

## Perspectives for treatment and prevention of PAH

The number of studies examining epigenetic alterations in PAH has been steadily increasing recently. These experimental and clinical studies have demonstrated that epigenetic processes, such as DNA methylation, ubiquitination, miRNAs-dependent gene regulation, and HDACs are related to PAH (Figure 1), as shown in different animal models. In addition, some reports have demonstrated that restoration of miRNA expression and HDACs inhibitors can be used to attenuate or reverse pathophysiological dysfunction of PAH. Despite the recent advances in the epigenetic field, the identification of a clinical epigenetic therapy with effective reversibility or cure for PAH is still a challenge for future research. A clinically relevant point raised by Wang and colleagues is that the majority of studies on animal models do not evaluate in depth the disadvantages or collateral effects provoked by epigenetic treatment (89), and initial preclinical studies with epigenetic modifiers have failed to show clinical significance. These issues should be the focus of future investigations.

**Figure 1.** Epigenetic mechanisms contributing to excessive proliferation and resistance to apoptosis of pulmonary artery smooth muscle cells (PASMCs) in pulmonary arterial hypertension (PAH) include: *i*) DNA methylation via DNA methyltransferases (DNMTs); *ii*) histone modifications, mainly methylation and acetylation, regulated by histone acetyltransferases (HATs) histone methyltransfereses (HMTs), histone deacetylases (HDACs), and histone demethylases (HDMs). Dysregulation of the ubiquitination process, as well as of microRNAs (miRNA, miR-) also participates in the pathogenesis of PAH. Epigenetic therapy based on DNMT inhibitors, HADAC inhibitors, proteasome inhibitors, and miR-RNA modulators are able to reduce the PASMCs proliferative state in PAH.

In addition, more studies examining the epigenetic pathway alterations underlying endothelial dysfunction will be necessary. In brief, it has been demonstrated that epigenetic factors, such as hypermethylation in HDAC4, HDAC5, and HDAC6 gene promoters, down-regulation in miR424/503, up-regulation of miR21, miR143, miR210, miR27a, and miR130/301, and upregulation of ion channels could display a potential function in molecular pathways alterations implicated in endothelial dysfunction in PAH (90).

Lastly, effective prevention of PAH needs to be investigated in future research. Experimental protocols examining the epigenetic process in the pre-pathological state of PAH will help to elucidate possible prevention strategies. For example, it is still unclear whether epigenetic modifications could be preceding the clinical manifestations of PAH. Monocrotaline-induced pulmonary arterial hypertension models in rodents have been shown to exhibit pathophysiological dysfunction after 28 days of intervention. Perhaps, future epigenetic experiments conducted at 14 days in these models will shed some light on the understanding of the pre-pathological epigenetic events before PAH.

## Conclusion

DNMT, HDAC, proteasome inhibitors, and up- or down-regulation of miRNAs can be useful as therapeutic targets in PAH treatment. Modulations of target epigenetic mechanisms are able to reduce the PASMCs proliferative state in PAH and consequently improve right ventricular systolic pressure and right ventricular hypertrophy.
